# Protective Effects of Total Flavonoids from *Lysimachia christinae* on Calcium Oxalate-Induced Oxidative Stress in a Renal Cell Line and Renal Tissue

**DOI:** 10.1155/2021/6667902

**Published:** 2021-09-20

**Authors:** Jian Wang, Jia-Jian Chen, Jia-Hao Huang, Bo-Dong Lv, Xiao-Jun Huang, Qing Hu, Jun Fu, Wen-Jie Huang, Ting-Ting Tao

**Affiliations:** ^1^The Second Clinical Medical College, Zhejiang Chinese Medical University, 310053 Hangzhou, China; ^2^Department of Urology, The Second Affiliated Hospital of Zhejiang Chinese Medical University, 310005 Hangzhou, China; ^3^Zhejiang Provincial Key Laboratory of Traditional Chinese Medicine, 310053 Hangzhou, China; ^4^Andrology Laboratory on Integration of Chinese and Western Medicine, Zhejiang Provincial Key Laboratory of Traditional Chinese Medicine, 310053 Hangzhou, China; ^5^Zhejiang Provincial Key Laboratory of Sexual function of Integrated Traditional Chinese and Western Medicine, 310053 Hangzhou, China

## Abstract

Oxidative stress (OS) in renal tubular epithelial cells (RTECs) is induced by calcium oxalate (CaOx) stones and plays an important role in the pathology of CaOx nephrolithiasis. The nuclear factor-E2-related factor 2 (Nrf2)/antioxidant response element (ARE) pathway is an important endogenous antioxidant pathway. Flavonoids are compounds with 2-phenylchromone as the basic mother nucleus and are natural antioxidant components of *Lysimachia christinae*. Our previous studies demonstrated that the total flavonoids from *L. christinae* (TFL) reduced calcium and oxalic acid concentrations in urine, thus inhibiting CaOx stone formation. We also showed that TFL can reduce OS in renal tissue. However, whether TFL inhibit the formation of CaOx stones through the Nrf2/ARE pathway requires further investigation. Here, we found that TFL protected against injury to a renal cell line and renal tissue, reduced CaOx-induced OS in renal tissue, and reduced CaOx crystal formation. In addition, TFL significantly increased nuclear Nrf2 and the expression of the downstream antioxidant genes heme oxygenase 1 (HO-1) and NAD(P)H quinone oxidoreductase 1 (NQO-1). Furthermore, TFL increased superoxide dismutase (SOD) activity and decreased the malondialdehyde (MDA) content, thereby alleviating OS in RTECs. Silencing Nrf2 expression blocked the protective effect of TFL on CaOx-induced OS. Taken together, our findings indicate that TFL reduce CaOx-induced OS in renal tissue by activating the Nrf2/ARE pathway.

## 1. Introduction

Calcium oxalate (CaOx) stones account for more than 70% of renal calculi [1]. The causes of urinary stones are extremely complex. It is generally believed that urinary stone formation is not caused by a single factor but a joint action of genetic, environmental, dietary, and metabolic factors [2, 3]. Several studies have shown that renal tubule epithelial cell (RTEC) injury may be a key factor causing the formation of renal calculi [4, 5]. RTEC injury leads to changes in the structure of the cell membrane. This provides an effective site for calcium salt crystal adhesion and promotes the deposition and aggregation of crystals into stones [6, 7]. Furthermore, RTECs exposed to high concentrations of oxalic acid or CaOx crystals can produce abundant reactive oxygen species (ROS) and have reduced superoxide dismutase (SOD) and catalase activities, which can cause oxidative stress (OS), even leading to RTEC apoptosis and death [8]. ROS-induced RTEC injury and subsequent OS are closely related to the formation of renal calculi and may even be an important initiating event. Therefore, we speculated that reducing OS in renal tissue may prevent the formation and recurrence of renal calculi.

OS is the result of an imbalance between intracellular pro-oxidant and antioxidant defense systems. When the intracellular antioxidant capacity is insufficient or weakened, OS occurs [9, 10]. Nuclear factor (NF)-E2-related factor 2 (Nrf2)/antioxidant response element (ARE) is an important endogenous anti-OS signaling pathway and is a major regulatory factor of antioxidant resistance [10, 11]. Several studies have shown that the absence of Nrf2, or functional damage to Nrf2, can aggravate OS, while Nrf2 activators can prevent kidney disease progression by protecting cells from oxidative damage [12, 13]. The Nrf2 activator dimethyl fumarate can alleviate calcium deposition and renal tissue injury induced by hyperoxaluria in rats and downregulate the expression of bone morphogenetic protein 2 and osteopontin [14].

Flavonoids are compounds with 2-phenylchromone as the basic mother nucleus. These molecules are important natural antioxidants and are the main active components in *Lysimachia christinae* [15, 16]. Indeed, flavonoids have high efficacy and low toxicity in the prevention and treatment of ROS-associated diseases. Some flavonoids act as antioxidants and Nrf2 activators, which activate the Nrf2 signaling pathway [17]. In vitro cell experiments showed that the total flavonoids from *L. christinae* (TFL) protected against cell damage induced by CaOx crystals. Our previous study demonstrated that TFL reduced calcium and oxalic acid concentrations in the urine, thus inhibiting CaOx stone formation [18]. We also confirmed that TFL can reduce OS in renal tissue [19]. Therefore, the specific mechanism underlying TFL inhibition of CaOx stone formation is worthy of further investigation.

Here, we investigated whether TFL reduced renal tissue OS induced by CaOx stone formation via Nrf2/ARE pathway activation. We hypothesized that Nrf2/ARE activation would prevent CaOx stone formation. We showed that TFL reduced OS in renal tissue induced by CaOx accumulation and reduced CaOx crystal formation. Importantly, we confirmed that TFL significantly increased the nuclear Nrf2 content and hemeoxygenase-1 (HO-1) and NAD(P)H quinone oxidoreductase 1 (NQO-1) protein expression in HK-2 cells treated with CaOx crystals. In addition, TFL treatment significantly increased SOD activity and decreased malondialdehyde (MDA) content in HK-2 cells, thereby reducing OS in RTECs. Silencing Nrf2 expression blocked the protective effect of TFL on CaOx-induced OS. Thus, TFL reduce CaOx-induced OS in renal tissue by activating the Nrf2/ARE pathway.

## 2. Materials and Methods

### 2.1. Reagents and Antibodies

TFL (power of *Lysimachia christinae* extract with content of 20% total flavonoids) were purchased from DASF Biotechnology Co. (Nanjing, China; catalog no. 180526A). Ethylene glycol (catalog no. 20181029) and ammonium chloride (catalog no. 2018030) were purchased from Sinopharm (Beijing, China). Calcium oxalate (catalog no. SJ0072CF88979), diphenyleneiodonium (catalog no. D2926), 3-(4,5-dimethylthiazol-2-yl)-2,5-diphenyltetrazolium bromide tetrazolium (MTT; catalog no. M2128), and dimethyl sulfoxide (catalog no. D5879) were obtained from Sigma-Aldrich (USA). Penicillin-streptomycin (catalog no. 15140-122) and fetal bovine serum (catalog no. 10099-141) were purchased from Gibco (USA). Antibodies against Nrf2 (batch no. ab62352), HO-1 (catalog no. ab69544), and NQO-1 (catalog no. ab34173) were obtained from Abcam (USA). Horseradish peroxidase-conjugated secondary antibodies were acquired from Bio-Rad (USA; catalog no. 172-6522). RIPA lysis solution (catalog no. P00138), tris buffer, bicinchoninic acid (BCA) protein assay (catalog no. P0012S), total superoxide dismutase (WST-8; catalog no. S0101) and lipid peroxidation MDA (catalog no. S0131) assays, and nuclear and cytoplasmic protein extraction kits (catalog no. P0027) were purchased from Beyotime (Shanghai, China). Polyvinylidene difluoride membranes were purchased from Millipore (USA; catalog no. IPVH00010). Annexin V-FITC/PI kits were purchased from Solarbio. Lipofectamine 2000 reagent was purchased from Thermo Fisher (USA; catalog no. 11668027).

### 2.2. Animal Experiments

All animal experiments were approved by the Animal Experimental Ethics Committee of Zhejiang Chinese Medical University. Fifty adult male Sprague-Dawley rats (250–300 g) were purchased from the Laboratory Animal Center of Zhejiang Chinese Medical University. All rats were housed in cages at 20 − 25°C and 40–60% humidity, under a 12-h light/dark cycle. Rats were weighed and divided randomly into five groups: normal control (NC); CaOx stone model (M), rats treated with 0.5% glycol and 2% ammonium chloride (1 mL/rat/d) in drinking water; CaOx stone model + low-dose TFL (LT) (62.5 mg/kg/d TFL); CaOx stone model + medium-dose TFL (MT) (125 mg/kg/d TFL); and CaOx stone model + high-dose TFL (HT) (250 mg/kg/d TFL). Each group was treated for 28 days. At the end of the experiment, the rats were weighed. After being anesthetized with intraperitoneal pentobarbital, the kidneys were quickly excised, weighed, fixed in 4% paraformaldehyde solution, frozen in liquid nitrogen, and stored at −80°C. Renal hypertrophy was assessed using the kidney/body weight ratio.

### 2.3. Histopathologic Scoring

Kidney cortex samples were fixed in 4% paraformaldehyde, embedded in paraffin, serially sectioned (4 *μ*m thickness), and stained with hematoxylin/eosin. Ten visual fields from each section were observed under a microscope at 100×  magnification. The degree of crystallization and renal tubular dilatation were scored for each visual field, and the average crystallization and dilation scores were calculated. The scoring criteria for crystallization were as follows: 0, no crystals; 1, few crystals (one or two per field); 2, moderate number of crystals (10–20 per field); and 3, high number of crystals (≥20 per field). Renal tubule dilation was scored as follows: 0, no obvious expansion; 1, scattered mild expansion; 2, extensive mild expansion, with scattered moderate expansion; 3: extensive moderate expansion, with scattered severe expansion; and 4: extensive severe expansion.

### 2.4. Small Interfering (si)RNA Transfection

SiRNA sequences targeting the Nrf2 gene, and scrambled siRNA negative controls, were purchased from Sangon Biotech (Shanghai, China). The Nrf2-siRNA sequence was 5′-GCCUGUAAGUCCUGGUCAUTT-3′, and the nonspecific negative control siRNA sequence was 5′-UUCUCCGAACGUGUCACGUTT-3′. Transient transfections were performed using the Lipofectamine 2000 transfection reagent.

### 2.5. Cell Culture

Human proximal tubular cells (HK-2 cells) were provided by the Laboratory Animal Center of Zhejiang Chinese Medical University (Hangzhou, China). The cells were maintained in Dulbecco's modified Eagle's medium containing 1 × penicillin-streptomycin and 10% fetal bovine serum at 37°C. The cells were subcultured with 0.25% trypsin when they reached 80% confluency. Cells in the logarithmic growth phase were harvested and seeded in 6-well plates until they reached 70–80% confluence. Then, HK-2 cells were divided into seven groups: (1) normal control (NC), (2) CaOx crystal model (M, HK-2 cells were treated with 2 mM CaOx crystal suspension), (3) M + TFL (HK-2 cells were treated with 2 mM CaOx crystal suspension and 50 *μ*g/mL TFL), (4) Nrf2 siRNA (HK-2 cells were transfected with NRF2-siRNA), (5) NC siRNA (HK-2 cells were transfected with control siRNA), (6) Nrf2 siRNA + M (HK-2 cells were transfected with NRF2-siRNA and then were treated with 2 mM CaOx crystal suspension), and (7) Nrf2 siRNA + M + TFL (50 *μ*g/mL).

### 2.6. Cell Viability Assay

Cell viability was determined using the 3-(4,5-dimethylthiazol-2-yl)-2,5-diphenyltetrazolium bromide (MTT) assay. Briefly, HK-2 cells in the logarithmic phase were seeded at 100 *μ*L per well in 96-well plates and incubated in an incubator at 37°C with 5% CO_2_. After treatment, 20 *μ*L of 5 mg/mL MTT was added to each well and the cells were incubated for 4 h at 37°C. The supernatant was discarded, and 150 *μ*L of dimethyl sulfoxide was added to each well. The mixture was gently shaken in a mini shaker at room temperature for 10 min. Absorbance at 490 nm was measured on a microplate reader (Molecular Devices, USA). The percent viability of treated cells was calculated using the formula:

(1) $$\begin{array}{c} \text{viablity}\left(\%\right)=\left(\frac{{\text{OD}}_{\text{treated}}-{\text{OD}}_{\text{blank}}}{\left({\text{OD}}_{\text{negative control}}-{\text{OD}}_{\text{blank}}\right)}\right)\times 100. \end{array}$$

### 2.7. Flow Cytometric Detection of Apoptosis

Apoptotic cell death was determined using the Annexin V-FITC/PI Apoptosis Kit according to the manufacturer's instructions. Cells were analyzed using flow cytometry.

### 2.8. Oxidative Stress

Renal MDA and total SOD levels of kidney tissue and HK-2 cells were determined using commercial kits to evaluate the degree of oxidative stress.

### 2.9. Western Blotting

Western blotting was performed to detect the expression of Nrf2, HO-1, and NQO-1. HK-2 cells were lysed in RIPA lysis buffer containing 1% phenylmethylsulfonyl fluoride and centrifuged at 12,000 rpm for 15 min at 4°C. The total protein concentration was determined using a BCA protein assay kit. Cell membrane proteins and nucleoproteins were extracted using a Cell Cytoplasmic Protein/Nucleoprotein Extraction kit. After denaturation, proteins were separated by sodium dodecyl sulfate-polyacrylamide gel electrophoresis and transferred to polyvinylidene difluoride membranes. After blocking with Tris buffer solution containing 5% nonfat milk for 1 h at 25 − 30°C, the membranes were incubated overnight at 4°C with primary antibodies against Nrf2, HO-1 and NQO-1. After thorough washing, the blots were incubated with a horseradish peroxidase-conjugated secondary antibody. Images were captured using an Odyssey two-color infrared laser imaging system (Li-Cor, Lincoln, NE, USA) and analyzed using Quantity One 1.62 software.

### 2.10. Statistical Analyses

All data were analyzed using SPSS 24.0 software. Normally distributed data are expressed as means ± SEM. Analysis of variance was used for multiple comparisons of the data followed by Fisher's post hoc least significant difference test. Tamhane's *T*2 tests were used for data with heterogeneous variances. Data that were not normally distributed are expressed as the median (M (range)), and the Wilcoxon rank sum test was used to compare these groups. *P* < 0.05 was considered statistically significant.

## 3. Result

### 3.1. CaOx Crystals Induce Apoptosis and Reduce the Viability of HK-2 Cells

HK-2 cells were treated with CaOx crystal suspensions (0.1, 0.25, 0.5, 1.0, 2.0, and 4.0 mM) for 24 h, and apoptosis was detected by flow cytometry. The percentage of cells undergoing apoptosis in response to 0, 0.1, 0.25, 0.5, 1.0, 2.0, and 4.0 mM CaOx treatment was 3.41 ± 0.78%, 8.48 ± 0.32%, 13.6 ± 0.57%, 21.2 ± 0.85%, 26.1 ± 0.76%, 35.4 ± 0.62%, and 45.4 ± 0.46%, respectively (Figure 1). The MTT assay showed that CaOx crystals decreased HK-2 cell viability in a concentration- and time-dependent manner (Figure 2).

### 3.2. TFL Protect HK-2 Cells from Damage Induced by CaOx Crystals

The percentages of cells undergoing apoptosis after 2 h pretreatment with 0, 10, 25, 50, and 125 *μ*g/mL TFL, followed by treatment with a 2 mM CaOx crystal suspension for 24 h, were 27.4 ± 5.00%, 24.4 ± 2.64%, 17.3 ± 2.34%, 13.7 ± 1.92%, and 12.3 ± 2.20%, respectively (Figure 3). Apoptosis significantly decreased after pretreatment with 25, 50, and 125 *μ*g/mL TFL compared with the control group (*P* < 0.01), but there was no significant difference between the 50 and 125 *μ*g/mL groups (*P* > 0.05). The MTT assay showed that TFL treatment mitigated the damage to HK-2 cells induced by CaOx crystals, while cell survival increased gradually with increasing concentrations of TFL (Figure 4). The survival of cells pretreated with 50 and 125 *μ*g/mL of TFL was significantly higher than that of the control group (*P* < 0.01 and *P* < 0.01, respectively), but there was no significant difference between these two groups (*P* > 0.05).

### 3.3. TFL Reduces CaOx Stone-Induced OS In Vitro and In Vivo

SOD activity in CaOx crystal-treated HK-2 cells was significantly lower (*P* < 0.01) than that in normal control HK-2 cells, and the MDA content was higher (*P* < 0.05) (Figure 5). This confirmed the presence of OS in CaOx crystal-treated HK-2 cells. After intervention with TFL, SOD activity was significantly increased (*P* < 0.01) and the MDA content was markedly decreased (*P* < 0.01)compared with the levels in CaOx crystal-treated HK-2 cells not exposed to TFL (Figure 5), indicating that TFL can reduce OS induced by CaOx crystals. In vivo experiments confirmed the in vitro results. As shown in Figure 6, SOD activity in the kidney tissue of CaOx stone model rats was significantly lower (*P* < 0.01) and the MDA content was higher (*P* < 0.05) than those in the kidney tissue of control rats. After intervention with moderate and high TFL doses, SOD activity was significantly increased and the MDA content was decreased (*P* < 0.05),compared with the levels in model rats.

### 3.4. TFL Increases the Nuclear Nrf2 Content and Downstream Antioxidant Gene Expression in CaOx Crystal-Induced HK-2 Cells

Western blotting data showed that there was no significant difference in the expression of total Nrf2 protein between HK-2 cells treated with CaOx crystals and normal cells (*P* > 0.05) (Figure 7). However, Nrf2 expression in nuclear extracts and HO-1 and NQO-1 expression were upregulated in CaOx crystal-treated HK-2 cells (Figure 7). After intervention with TFL, nuclear Nrf2, HO-1, and NQO-1 expressions were further increased and intracellular Nrf2 expression was decreased (Figure 7), indicating that TFL increase the nuclear Nrf2 content and downstream antioxidant gene expression.

### 3.5. Nrf2/ARE Pathway Is Downregulated in HK-2 Cells after Nrf2 siRNA Treatment

We first evaluated the Nrf2/ARE pathway by inactivating it with Nrf2 siRNA. After Nrf2 siRNA treatment, total Nrf2, intracellular Nrf2, nuclear Nrf2, HO-1, and NQO-1 expressions were efficiently decreased (*P* < 0.01) in HK-2 cells compared with NC Nrf2 siRNA treatment (Figure 8). Along with decreasing Nrf2 levels, Nrf2 siRNA markedly reduced the HO-1 and NQO-1 protein levels (*P* < 0.01) (Figure 8), indicating that we could effectively silence the expression of Nrf2 in cells and affect the expression of downstream genes by siRNA treatment. Importantly, Nrf2 siRNA treatment reversed the upregulated expression of nuclear Nrf2, HO-1, and NQO-1 induced by CaOx crystals in HK-2 cells (Figure 7). The levels were even lower than those in the normal control group (*p* < 0.01). Furthermore, after Nrf2 siRNA treatment, TFL did not show any effect on the expression of nuclear Nrf2, HO-1, and NQO-1 in CaOx crystal-treated HK-2 cells (Figure 7).

### 3.6. Nrf2/ARE Pathway Mediates the Effect of TFL on OS

TFL treatment significantly increased SOD activity and significantly reduced the MDA content in HK-2 cells treated with CaOx crystals (Figure 5). TFL also increased nuclear Nrf2, HO-1, and NQO-1 expressions (Figure 7). However, Nrf2 siRNA treatment reversed the upregulated expression of nuclear Nrf2, HO-1, and NQO-1, induced by TFL in CaOx crystal-treated HK-2 cells (Figure 8). And as shown in Figure 5, Nrf2 siRNA treatment markedly decreased SOD activity (*P* < 0.01) and increased the MDA content (*P* < 0.01) in CaOx crystal-treated HK-2 cells exposed to TFL. These results were significantly different from the results in CaOx crystal-treated HK-2 cells treated with TFL and were not different from the results in HK-2 cells treated with Nrf2 siRNA and CaOx alone (*P* > 0.05), indicating that there was no significant effect of TFL treatment on CaOx crystal-induced OS after Nrf2 siRNA treatment.

### 3.7. TFL Inhibit the Formation of Renal Calculi in a CaOx Stone Rat Model

As shown in Table 1, CaOx stone model rats exhibited diminished body weight and a higher kidney weight/body weight ratio, which indicates kidney hypertrophy compared with normal rats. Hematoxylin/eosin staining showed broadly dilated kidney tubules and crystal deposition in the renal tubule lumen of CaOx stone model rats (Figure 9); the crystallization score was 2.30 ± 0.26, and the renal tubule dilation score was 3 (Table 1). These scores were significantly higher than those in the normal control group, which suggests that the CaOx stone rat model was successfully established. Rats in the high-dose TFL treatment group showed a reduced kidney weight/body weight ratio, a low degree of crystal formation, and a lower degree of renal tubule dilation than did CaOx stone model rats (Table 1). However, treatment with low- and medium-dose TFL did not show a significant effect.

## 4. Discussion

The mechanism of renal calculus formation is very complex. However, an increasing number of studies have shown that RTEC injury is an important cause of renal calculus formation [20]. Thus, it is important to study the interaction between CaOx crystals and RTECs to understand the formation and pathogenesis of renal calculi. When CaOx crystals interact with RTECs, they cause oxidative damage, which leads to cell death and damage to nearby cells [21]. The damaged cells gradually become fragments, which then become nucleation centers that allow further crystal aggregation, ultimately causing the cascade reaction for stone formation. Farell et al. [22] summarized the pathophysiological process of renal calculus formation. Specifically, CaOx crystals act on RTECs and activate NADPH oxidase. The abnormal increase in OS leads to mitochondrial death, caspase-3 activation, cell damage, structural changes in membrane phosphatidylserine, and renal crystal adhesion.

The present study demonstrated that varying concentrations of CaOx crystal damages HK-2 cells. Cell viability was negatively correlated with the concentration and time of exposure, the rate of apoptosis increased with CaOx crystal concentration, and exposure to CaOx crystal significantly decreased SOD activity and increased MDA content in HK-2 cells. Treating rats with 0.5% glycol and 2% ammonium chloride also decreased SOD activity and increased renal MDA levels. SOD is a type of antioxidant enzyme, which can transform superoxide anions into H_2_O_2_ to play a role in antioxidant stress. MDA is a stable end product of OS that indirectly reflects the production of OS. Therefore, SOD activity and MDA content are often used to evaluate OS in vivo. These results suggest that CaOx calculi induce OS in HK-2 cells and renal tissue.

During OS, the accumulation of free radicals overwhelms the capacity of the endogenous antioxidant system to effectively neutralize excessive ROS, resulting in cell damage and dysfunction [23]. Therefore, it is believed that the provision of exogenous antioxidants might alleviate OS. Although such strategies are effective in treating OS in vitro and in in vivo animal models [24, 25], they are often ineffective in long-term clinical trials [26]. This could be due to the water-soluble nature of most exogenous antioxidants, which thus often require administration in large dosages to achieve the desired effect. However, excessive dosing might increase the risk of adverse effects and toxicity [27] and could interfere with processes reliant on physiological levels of ROS [28]. Therefore, a more effective novel approach to treat oxidative stress-related disorders might be the activation of endogenous antioxidant stress-response pathways or enhancement of the antioxidant and anti-inflammatory effects of natural antioxidants.

Flavonoids, an important class of natural antioxidants, exhibit a variety of biological activities, comprise an important class of natural antioxidants (involved in processes including the modulation of cellular functions), can act on the antioxidant signaling pathways in cells, activate transcription factors, and have initiation start sites for downstream gene expression. This contributes to the maintenance of human cells and tissues in a state of redox balance, thereby preserving the physiological normal functions of the body and preventing the occurrence of diseases. Zhou [17] extracted a variety of flavonoids from *Cinnamomum camphora* and demonstrated that they could activate the Nrf2 signaling pathway. Moreover, flavonoids exhibit high efficacy and low toxicity in the prevention and treatment of OS-related disorders [29]. Many medicinal plants and their derivatives contain flavonoids. For example, the TFL complement of *L. christinae* represents the main active constituents responsible for its therapeutic effects. This TFL complement exerts antioxidant, urinary calculi-preventive, diuretic, cardioprotective, cerebrovascular protective, anti-inflammatory, and analgesic effects, with almost no associated acute toxicity [30].

This study confirmed that exposing HK-2 cells undergoing CaOx-induced OS to TFL significantly increased SOD activity and decreased MDA levels, suggesting that TFL oppose CaOx crystal-induced OS. This effect was recapitulated in the rat model; after intervention with a certain dose of TFL, SOD activity was significantly increased and the MDA content was decreased compared with the levels in model rats. Moreover, rats in the high-dose TFL treatment group also showed a reduced kidney weight/body weight ratio, a low degree of crystal formation, and a lower degree of renal tubule dilation than CaOx stone model rats, which means that TFL decreased CaOx crystallization and renal tissue damage. These observations indicate that TFL-mediated inhibition of CaOx calculus formation might be closely associated with decreased renal OS. To elucidate the mechanisms underlying this phenomenon, we investigated whether the protective antioxidant effects of TFL on renal tissue are mediated by Nrf2/ARE pathway modulation, thereby preventing renal calculus formation.

The Nrf2/ARE pathway is an important endogenous anti-OS pathway used for defense against oxidative and electrophilic stress. Nrf2 has antioxidant effects and is an important target for the prevention and treatment of OS-related diseases [10], thereby maintaining the stability of the intracellular environment and immune surveillance. Previous studies have shown that some flavonoids are activators of Nrf2 and exert antioxidant effects by activating the Nrf2 signaling pathway [17].

After confirming that TFL reduced OS in renal tissue using in vitro and in vivo CaOx stone models, we investigated the effect of TFL on the Nrf2-ARE pathway. In vitro experiments revealed that after HK-2 cells were treated with CaOx crystals, activated Nrf2 was recruited to the nucleus. Nrf2 binding with the ARE initiates downstream gene transcription, thereby upregulating HO-1 and NQO-1 expression and activating an anti-OS reaction. TFL treatment further increased nuclear Nrf2 content and increased HO-1 and NQO-1 protein expression in HK-2 cells treated with CaOx. In addition, TFL treatment significantly increased SOD activity and decreased MDA content in CaOx crystal-treated HK-2 cells. These results confirmed the effect of TFL on the Nrf2-ARE pathway and indicated that the protective effect of TFL on OS might be mediated by activation of the Nrf2/ARE pathway.

Based on these results, Nrf2 siRNA treatment was undertaken to uncover whether the protective effects of TFL on OS involved activating the Nrf2/ARE pathway. SiRNA, also known as a silent RNA and noncoding RNA, is a small RNA fragment with a specific length and sequence that can combine with the mRNA expressed by genes in the form of a single strand, inducing the degradation of this mRNA and resulting in the silencing of target gene expression [31]. Transfecting Nrf2 siRNA into HK-2 cells caused the expression of Nrf2, HO-1, and NQO-1 to decrease significantly, verifying that the transfection was successful. Furthermore, Nrf2 siRNA treatment significantly prevented TFL-induced nuclear Nrf2, HO-1, and NQO-1 upregulation in CaOx-treated HK-2 cells. Nrf2 siRNA treatment also markedly prevented the effect of TFL on increasing SOD activity and decreasing MDA content in CaOx-treated HK-2 cells. This indicates that there was no effect of TFL on CaOx crystal-induced OS after Nrf2 siRNA treatment. Thus, it is suggested that the protective effect of TFL on CaOx-induced OS in renal tissue is closely related to the Nrf2/ARE pathway.

## 5. Conclusion

Taken together, our findings indicate that TFL increased nuclear Nrf2, HO-1, and NQO-1 expressions and SOD activity in CaOx-treated HK-2 cells and rat models. Furthermore, TFL decreased the MDA content and reduced CaOx-induced OS, thereby decreasing RTEC apoptosis. Overall, TFL prevented CaOx stone formation in vivo and in vitro. These results illustrate that the protective effect of TFL on OS induced by CaOx is closely associated with the Nrf2/ARE pathway. Thus, we have clarified the mechanisms responsible for the effects of TFL in the prevention and treatment of renal calculi.

## Figures and Tables

**Figure 1:** Effects of different concentrations of CaOx on HK-2 cell apoptosis.

**Figure 2:** Effects of different concentrations and treatment time of CaOx crystals on the viability of HK-2 cells. ^*∗*^*P* < 0.05, ^∗∗^*P* < 0.01 vs 0 mM oxalate group.

**Figure 3:** Effects of different concentrations of TFL on HK-2 cell apoptosis induced by CaOx crystals.

**Figure 4:** Effect of different concentrations of TFL on the viability of CaOx crystals-induced HK-2 cells. ^*∗*^*P* < 0.05, ^∗∗^*P* < 0.01 vs 0 mM oxalate group.

**Figure 5:** Effect of TFL and Nrf2 siRNA on CaOx stone-induced OS in HK-2 cells. (a) SOD activity in HK-2 cells. (b) MDA content in HK-2 cells. ^*∗*^*P* < 0.05 and ^∗∗^*P* < 0.01 vs the NC group. ^#^*P* < 0.05, ^##^*P* < 0.01 vs M group. ^Δ^*P* < 0.05, ^ΔΔ^*P* < 0.01 vs M + TFL group.

**Figure 6:** Effect of TFL on CaOx stone-induced OS in renal tissue. (a) SOD activity in renal tissue. (b) MDA content in renal tissue. ^*∗*^*P* < 0.05, ^∗∗^*P* < 0.01 vs NC group. ^#^*P* < 0.05, ^##^*P* < 0.01 vs M group.

**Figure 7:** Effect of TFL and Nrf2 siRNA on the expression of Nrf2, HO-1, and NQO-1 in CaOx-treated HK-2 cells. (a) Western blot analyses showing the protein expression levels of Nrf2, HO-1, and NQO-1 after treatment with CaOx, TFL, and Nrf2 siRNA. (b) Relative density of total Nrf2, intracellular Nrf2, nuclear Nrf2, HO-1, and NQO-1 expression with *β*-actin as the loading control. Values are presented as means ± SEM. ^*∗*^*P* < 0.05, ^∗∗^*P* < 0.01 vs NC group. ^#^*P* < 0.05, ^##^*P* < 0.01 vs M group.

**Figure 8:** Effect of Nrf2 siRNA on the expression of Nrf2, HO-1, and NQO-1 in HK-2 cells. (a) Western blot analyses showing the protein expression levels of Nrf2, HO-1, and NQO-1 after transfecting Nrf2 siRNA into HK-2 cells. (b) Relative density of total Nrf2, intracellular Nrf2, nuclear Nrf2, HO-1, and NQO-1 expression with *β*-actin as the loading control. Values are presented as means ± SEM. ^*∗*^*P* < 0.05, ^∗∗^*P* < 0.01.

**Figure 9:** Representative hematoxylin/eosin staining of kidney tubules of the normal control (NC), CaOx stone model M, M + low-dose TFL (LT), M + medium-dose TFL (MT), and M + high-dose TFL (HT) groups (100 × magnification).

**Table 1:** Effect of TFL on the renal tissue of CaOx stone model rats.

Parameters	NC	M	LT	MT	HT
BW loss (g)	7.00 ± 13.65	45.5 ± 24.2^∗∗^	32.0 ± 19.2^∗∗^	31.5 ± 9.8^∗∗^	28.8 ± 20.8^∗∗#^
KW (g)	1.89 ± 0.29	2.64 ± 0.86^∗∗^	2.65 ± 0.69^∗∗^	2.58 ± 0.70^*∗*^	2.15 ± 0.28
KW/BW (%)	0.69 ± 0.09	1.07 ± 0.40^∗∗^	1.09 ± 0.26^∗∗^	0.95 ± 0.21^∗∗^	0.84 ± 0.10^#^
SCD	0.50 ± 0.22	2.30 ± 0.26^∗∗^	2.00 ± 0.26^∗∗^	2.00 ± 0.21^∗∗^	1.50 ± 0.22^∗∗#^
SRTDD	0 (0–)	3 (1–4)^∗∗^	3 (1–4)^∗∗^	3 (1–4)^∗∗^	2 (1–3)^∗∗#^

SRTDD data are presented as medians (range). All other data are presented as means ± SEM. KW, kidney weight; BW, body weight; SCD, score of crystallization degree; SRTDD, score of renal tubule dilatation degree. ^*∗*^*P* < 0.05 and ^∗∗^*P* < 0.01 vs Group *A*. ^#^*P* < 0.05 and ^##^*P* < 0.01 vs Group *B*.

## Data Availability

The data used and analyzed in the present article are available from the corresponding author on reasonable request.

## References

[1] Lieske J. C., Rule A. D., Krambeck A. E. (2014). Stone composition as a function of age and sex. *Clinical Journal of the American Society of Nephrology*.

[2] Attanasio M. (2011). The genetic components of idiopathic nephrolithiasis. *Pediatric Nephrology*.

[3] Parvin M., Shakhssalim N., Basiri A. (2011). The most important metabolic risk factors in recurrent urinary stone formers. *Urology Journal*.

[4] Khan S. R. (2006). Renal tubular damage/dysfunction: key to the formation of kidney stones. *Urological Research*.

[5] Tsujihata M. (2008). Mechanism of calcium oxalate renal stone formation and renal tubular cell injury. *International Journal of Urology*.

[6] Khan S. R., Canales B. K. (2015). Unified theory on the pathogenesis of Randall’s plaques and plugs. *Urolithiasis*.

[7] Fasano J. M., Khan S. R. (2001). Intratubular crystallization of calcium oxalate in the presence of membrane vesicles: an in vitro study. *Kidney International*.

[8] Thamilselvan S., Byer K. J., Hackett R. L., Khan S. R. (2000). Free radical scavengers, catalase and superoxide dismutase provide protection from oxalate-associated injury to LLC-PK1 and MDCK cells. *The Journal of Urology*.

[9] Poljsak B., Šuput D., Milisav I. (2013). Achieving the balance between ROS and antioxidants: when to use the synthetic antioxidants. *Oxidative medicine and cellular longevity*.

[10] Abed D. A., Goldstein M., Albanyan H., Jin H., Hu L. (2015). Discovery of direct inhibitors of Keap1-Nrf2 protein-protein interaction as potential therapeutic and preventive agents. *Acta Pharmaceutica Sinica B*.

[11] Pajares M., Cuadrado A., Rojo A. I. (2017). Modulation of proteostasis by transcription factor NRF2 and impact in neurodegenerative diseases. *Redox biology*.

[12] Frijhoff J., Winyard P. G., Zarkovic N. (2015). Clinical relevance of biomarkers of oxidative stress. *Antioxidants & Redox Signaling*.

[13] Ratliff B. B., Abdulmahdi W., Pawar R., Wolin M. S. (2016). Oxidant mechanisms in renal injury and disease. *Antioxidants & Redox Signaling*.

[14] Zhu J., Wang Q., Li C. (2019). Inhibiting inflammation and modulating oxidative stress in oxalate-induced nephrolithiasis with the Nrf2 activator dimethyl fumarate. *Free Radical Biology & Medicine*.

[15] Wang Z. J., Dai B., Wang F. M. (2008). Microwave technique extraction and determination of total flavonoids and polysaccharides in lysimach christinae hance. *Chinese Journal of Modern Applied Pharmacy*.

[16] Wu N.-H., Ke Z.-Q., Wu S. (2018). Evaluation of the antioxidant and endothelial protective effects of Lysimachia christinae Hance (Jin Qian Cao) extract fractions. *BMC Complementary and Alternative Medicine*.

[17] Zhou M. X. (2018). *Investigation on Natural Antioxidants Targeting Nrf2 Signaling Pathway*.

[18] Tao T. T., Lv B. D., Huang X. J., Fu J., Ma Y. F. (2020). Study on the total flavone extract of lysimachia on calcium oxalate stone formation in rats. *China Modern Doctor*.

[19] Tao T. T., Zhao F., Ye M. Y., Lv B. D., Fu J. (2020). Effect of total flavonoids from Christina Loosestrife (*Lysimachia Christinae*) on Osteopontin expression in renal tissue of calcium oxalate stone model rats. *Zhejiang Journal of Integrated Traditional Chinese and Western Medicine*.

[20] Narula S., Tandon S., Singh S. K., Tandon C. (2016). Kidney stone matrix proteins ameliorate calcium oxalate monohydrate induced apoptotic injury to renal epithelial cells. *Life Sciences*.

[21] Oliveira L. C. B. P., Queiroz M. F., Fidelis G. P. (2020). Antioxidant sulfated polysaccharide from edible red seaweed is an inhibitor of calcium oxalate crystal formation. *Molecules (Basel, Switzerland)*.

[22] Farell G., Huang E., Kim S. Y., Horstkorte R., Lieske J. C. (2004). Modulation of proliferating renal epithelial cell affinity for calcium oxalate monohydrate crystals. *Journal of the American Society of Nephrology*.

[23] Schrag M., Mueller C., Zabel M. (2013). Oxidative stress in blood in Alzheimer’s disease and mild cognitive impairment: a meta-analysis. *Neurobiology of Disease*.

[24] Karbach S., Wenzel P., Waisman A., Munzel T., Daiber A. (2014). ENOS uncoupling in cardiovascular diseases-the role of oxidative stress and inflammation. *Current Pharmaceutical Design*.

[25] Nezis I. P., Stenmark H. (2012). p62 at the interface of autophagy, oxidative stress signaling, and cancer. *Antioxidants & Redox Signaling*.

[26] Schmidt H. H. H. W., Stocker R., Vollbracht C. (2015). Antioxidants in translational medicine. *Antioxidants & Redox Signaling*.

[27] Moosmann B., Behl C. (2002). Antioxidants as treatment for neurodegenerative disorders. *Expert Opinion on Investigational Drugs*.

[28] Sedeek M., Nasrallah R., Touyz R. M., Hébert R. L. (2013). NADPH oxidases, reactive oxygen species, and the kidney: friend and foe. *Journal of the American Society of Nephrology*.

[29] Kozłowska A., Szostak-Wegierek D. (2019). Flavonoids--food sources and health benefits. *Roczniki Panstwowego Zakladu Higieny*.

[30] Zhang Z., Zhong Q., Zhou B. (2019). Research progress on extraction methods and pharmacological action of total flavonoids from Desmodium styracifolium. *Chinese Medicine Modern Distance Education of China*.

[31] Crooke S. T., Witztum J. L., Bennett C. F., Baker B. F. (2019). RNA-targeted therapeutics. *Cell Metabolism*.

[32] Wang J., Chen J. J., Huang J. H. (2020). Protective effects of total flavonoids from *Lysimachia Christinae* on calcium oxalate-induced oxidative stress in a renal cell line and renal tissue. https://www.researchsquare.com/article/rs-132214/v1.

